# The Effect of the Duckett procedure on the Outcome and Prognosis of Children with Suburethral Cleft

**DOI:** 10.1155/2022/7444104

**Published:** 2022-06-28

**Authors:** Hongqiong Geng, Shigang Cheng, Xinghai Yang, Yanqin Huang

**Affiliations:** Department of Surgery, Hubei Maternal and Child Health Care Hospital, Tongji Medical College, Huazhong University of Science and Technology, Wuhan 430070, China

## Abstract

**Background:**

Hypospadias is one of the most common malformations of the male genitourinary system. In recent years, the incidence of hypospadias is increasing year by year, which seriously affects normal urination and sexual function. Repairing hypospadias has always been a challenge in paediatric urology, requiring a variety of surgical techniques and science and art that requires intensive study. Despite the availability of over 300 surgical procedures and continuous improvement, there is still a high level of surgical complications. It is crucial to choose an appropriate and effective surgical method for the treatment of hypospadias.

**Aims:**

This study aimed to investigate the outcome and prognosis of children with hypospadias, using transverse cut foreskin island flap coiled urethroplasty (the Duckett procedure).

**Materials and Methods:**

A retrospective study was conducted on 100 children with hypospadias who underwent surgery in our hospital from December 2018 to December 2021. Based on the degree of hypospadias and the degree of penile curvature both in line with the Duckett procedure, the comparison group was treated with a one-stage Duckett procedure and the treatment group was treated with a staged Duckett procedure. The differences in the surgical condition, inflammatory factor levels, and complications between the two groups of children were observed and compared.

**Results:**

The length of hospital stay and VAS score in the treatment group were significantly lower than those in the control group, and the operation time and intraoperative bleeding were higher than those in the control group, with a statistical significance (*P* < 0.05). The success rate of one operation was higher than that of the comparison group, but the statistical comparison was not statistically significant (*P* > 0.05). There was no statistically significant difference in the inflammatory response between the two groups before surgery (*P* > 0.05), while the difference in CRP, IL-6, and calcitoninogen between the two groups after surgery was significant and lower in the comparison group than in the treatment group, which was statistically significant (*P* < 0.05). The clinical outcome of the children in both groups showed that the excellent rate of 92.00% in the treatment group was significantly higher than that of 74.00% in the comparison group, while the incidence of complications was significantly lower than that of the comparison group, and the difference was statistically significant (*P* < 0.05). Complications in children with poor surgical outcomes in both groups occurred mainly, early urethral stricture and cured by urethral dilatation or condition without improvement cured by urethrotomy.

**Conclusion:**

A comparative study of hypospadias treated with the staged Duckett procedure was more effective in relieving postoperative pain and inflammatory reactions in children, reducing postoperative complications and improving healing efficiency, providing some reference value for hypospadias surgery.

## 1. Introduction 

Hypospadias is a deformity of the external genitalia in which the urethral sulcus is not fully fused to the distal glans due to embryonic development disorders. The incidence is about 0.3% and the number of affected children is increasing year by year, which seriously affects the reproductive system of the affected children [1, 2]. At present, the clinical treatment of hypospadias is mostly urethroplasty, but different surgical methods have different effects on children, and there is no unified standard for clinical treatment [3]. There are many different types of urethroplasty, the most commonly used being the Duckett procedure [4]. Because of its ability to completely correct hypospadias as well as reconstruct the urethra in one stage and the aesthetic appearance of the penis after surgery, the Duckett procedure remains indispensable for cases with significantly combined hypospadias [5]. However, there is a high rate of complications associated with the one-stage Duckett procedure to repair severe hypospadias, and if penile appearance is sacrificed in order to reluctantly reconstruct the urethra in one stage, this may result in residual hypospadias and penile scar contracture, making reoperation difficult and postoperative results poor. Therefore, a planned staging surgery may be the right option in some cases with specific anatomical conditions. A complete correction of the penile curvature of heavy hypospadias is achieved by the first-stage surgery, with partial reconstruction of the new urethra without affecting the appearance of the penis, followed by reconstruction of the remaining urethra by the second-stage surgery [6]. Active stage surgery with segmental urethroplasty not only reduces the difficulty of the surgery, but also reduces the risk of postoperative complications and the difficulty of perioperative care for the child, and the emotional stress of the parents is significantly reduced. Based on this, we have conducted some exploration to investigate the effects of the staged Duckett procedure treatment on the outcome and prognosis of children with hypospadias, and the findings are now reported as follows.

## 2. Material and Methods

### 2.1. Research Object

According to the formula of cross-sectional survey sample size: *n*=(*t*_*a*_)^2^*PQ*/*d*^2^, *n* is the sample size, P is the prevalence of hypospadias, *Q* = 1 − *P*, *d* is the permissible error. *a* = 0.05, and *t*_*a*_ = 1.96. The minimum sample size of this study is 80 cases, and the actual sample size of this study is 100 cases; according to the degree of hypospadias and the degree of penile curvature, the patients are divided into the comparison group and the treatment group. Due to transfer, new crown epidemic, lost visits, etc., 5 cases were shed from each group ultimately leaving 50 cases each in each group. The indications for the staged Duckett surgery were as follows: (1) narrow penile head (diameter ≤ 1.2 M), penile dysplasia, and inability to achieve urethral orthodontic opening in the first stage of surgery; (2) severe hypospadias of the penis due to fibrous scar contracture of the urethral plate, which requires cutting off the urethral plate in order to fully straighten the penis and at the same time causing defects in the long segment of the urethra; (3) insufficient local skin material or poor development, making it difficult to perform urethroplasty and repair the (4) where the surgeon is not skilled or experienced enough to complete a one-stage Duckett repair. The correct choice of procedure will significantly reduce the incidence of postoperative complications such as urethral fistula or urethral stricture, thus increasing the success rate of the procedure.

### 2.2. Exclusion Criteria

#### 2.2.1. Inclusion Criteria and Exclusion Criteria

Inclusion criteria were as follows: (i) all the children in this study met the diagnostic criteria for hypospadias as defined by the expert consensus on hypospadias [7], and the patients had preserved urethral plates and noncircumcised tubes; (ii) children aged <14 years with moderate to severe hypospadias, who were compliant and gave informed consent; (iii) all were first-time urethroplasty patients. Exclusion criteria were as follows: (i) those aged ≥14 years who are contraindicated for this trial; (ii) those with combined urinary tract infections; (iii) those with other hypospadias, and those with previous severe cardiovascular disease, hypertension, coagulation abnormalities, diabetes mellitus, hepatitis, tuberculosis, or who are unsuitable for this study due to other factors.

### 2.3. Methods

In this case, the comparison group was treated with a one-stage Duckett procedure, i.e., correction of the inferior penile curvature. the foreskin was first circumcised at a distance of 0.5–1 cm from the coronal sulcus, while the urethral plate was transected. The foreskin is then deflowered, the penile skin is freed on the superficial side of the white membrane to the root of the penis, and the ventral fibrous band is freed and loosened to correct the curved deformity. If this is not completely corrected, the leucorrhoea is folded below the vascular nerve bundle on the dorsal side of the penis. Finally, an artificial erection test is performed to confirm complete correction of the hypospadias. Reconstruction of the urethra is performed as follows: the proximal urethral dysplastic tissue is first excised to the plane of the good urethral cavernous tissue and trimmed to a spatulate shape, and the proximal urethra is fixed with a 6-0 absorbable thread in the white membrane immediately adjacent to the penile shaft. The dorsal foreskin of the penis is then circumcised, an inner plate equivalent to the length and appropriate width of the defective urethra is measured, its corners are drawn with fine silk thread, a superficial transverse incision is made at the junction of the inner and outer plates and the superficial fascia is cut open with ophthalmic shears and its level maintained, and the vascular tip is freed proximally and laterally to the root of the penis. The flap is then turned ventrally and parallel to the penile thousand via the lateral side of the penis and the tipped foreskin flap is closed with interrupted 6-0 absorbable sutures, with the proximal end anastomosed to the trimmed urethral orifice and the sutures knotted out. Continuous full sutures are placed to form a new urethra. At the same time, the coronal sulcus of the penile head is dissected close to the superficial surface of the white membrane to form a tunnel of suitable calibre for the head of the penis. The proximal end of the new urethra is obliquely anastomosed to the external orifice of the original urethra. Finally, a multilateral perforated silicone stent tube of appropriate calibre is left in the urethra. Care should be taken when fixing the skin tube to the white membrane of the penis to keep the sutured edge of the skin tube as ventral as possible to the corpus cavernosum and to cover the urethral anastomosis with a portion of tissue from the vascular tip. Penile dermoplasty was performed as follows: The dorsal foreskin is cut medially to form a butterfly flap and transferred to the ventral side, with a Z-shaped suture covering the ventral penile skin defect.

The treatment group underwent a staged Duckett procedure, i.e., hypospadias correction. The incision design differed from the staged procedure as follows: the incision in the staged procedure was circumcised at the same time as the original external urethral opening in order to free the proximal urethra to straighten the penis and trim the external urethral opening for the anastomosis. In contrast, the staged incision is simply a transection of the urethral plate and circumcision of the foreskin without dissection to free the proximal urethra and trim the original urethral orifice. The rest of the procedure, such as circumcision, release of the ventral fibrous band, folding of the white membrane below the dorsal vascular nerve bundle of the penis, and the artificial erection test, are the same as those in the first stage. Reconstruction of a part of the urethra was performed as follows: firstly, as this procedure only anastomoses the posterior wall of the urethra, the original external urethral opening does not need to be trimmed to a spatulate shape. Second, the width of the dorsal foreskin island flap is the same as that in the first stage, but in some cases, the length may be limited by the material of the foreskin itself and may not match the length of the defective urethra; therefore, priority can only be given to the coverage of the remaining foreskin at the expense of the length of the island flap. The freeing of the island flap, the covering of the vascular tip, the new urethroplasty after the island flap transfer, the external urethroplasty, and the posterior urethral wall anastomosis are all the same as in the first stage. The main difference between this procedure and the first stage is the anastomosis of the anterior and lateral walls of the urethra. The proximal end of the new urethra is anastomosed to the posterior wall of the original urethral orifice, starting from the middle of the posterior wall of the anastomosis and reconstructing only about one-half to two-thirds of the anastomosis, keeping the triangular flap of the anterior wall of the new urethra sutured to the transfer flap on both sides of the foreskin and leaving the anterior wall of the urethral orifice open. Penile dermoplasty was performed as follows: the procedure is essentially the same as the first stage, except that when the new urethra is shorter than the length of the urethral defect, the dorsal foreskin is transferred and inserted between the posterior wall of the new urethra and the posterior wall of the original external urethral opening. A second operation is performed at around 9 months after the first operation, and depending on the length of the proximal urethral defect, when the defect is greater than 0.5 cm and less than 1 cm, a urethral fistula is repaired with a fascial flap of tissue to cover it. When the length of the defect is greater than 1 cm, TIP and Duplay are chosen for repair. Some cases with severe combined penile scrotal transposition are corrected at the second stage of surgery. In the early cases, routine urethral dilatation was performed at about 1 month after the first surgery in about 8 children, but no urethral contracture or adhesions were found, so routine urethral dilatation was not performed in any of the 24 children in the later cases.

### 2.4. Observation Indicators

In both the groups, bipolar electrocoagulation was used for haemostasis, micro instrumentation, and 6–0 absorbable sutures were used for closure. The new urethra was treated with an F6 or F8 silicone urethral balloon as a stent tube and no conventional cystostomy was performed in either group. The outer elastic bandage and middle mesh gauze were changed every 2–3 days after surgery, the outer elastic bandage and middle mesh gauze were removed in 6–7 days, the inner dressing was removed in 8–9 days, and the urinary catheter was removed in 12–14 days. The children were discharged after observation of no difficulty in urination, effort to urinate, and other discomforts 3. Cure criteria were as follows: urethral orifice located in the positive position of the head of the penis, complete correction of the downward curvature of the penis, near-normal appearance of the penis, ability to stand and urinate normally, no complications such as urinary fistula, urethral stricture, and urethral diverticulum. Case follow-ups were performed by telephone and outpatient in both the groups, based on the cut-off time obtained from the date of surgery to the last follow-up visit, and the cut-off date for both groups was 10 March 2022. (i) Analysis of the surgical situation was as follows: the intraoperative and postoperative time of the child's hospital stay, duration of surgery, VAS score, intraoperative bleeding, and success rate of one-stage surgery were recorded. (ii) Levels of inflammatory factors were as follows: inflammation-related indexes, i.e., C-reactive protein (CRP), interleukin-6 (IL-6), and calcitoninogen levels, were measured before and after surgery in both groups using immunoassays. (iii) clinical outcome was evaluated. Excellent was defined as penis straightening, normal urination, and patency; good was defined as penis straightening, normal urination, and complications without reoperation; poor was defined as penis not straightening, unable to urinate normally, or requiring reoperation.

### 2.5. Statistical Analysis

All statistical data in this study were input into Excel software by the first author and corresponding author, and the data were processed by SPSS25.0. Repeated measures analysis of variance between groups was used to measure the measurement expressed as mean ± standard deviation (*X* ± *S*). Count data were expressed as percentage (%) and tested by the *χ*^2^ test. Univariate and logistic multivariate regression analyses were used to compare the influencing factors, and the risk factors with significant differences were screened. Univariate and logistic multivariate regression analyses were used to compare the influencing factors, and the risk factors with obvious differences were screened. The statistical significance was *P* < 0.05.

## 3. Results

### 3.1. Comparison of General Information

The general data include age, body mass index, urethral plate width, and suburethral cleft case typing were compared between the two groups and there was no statistical significance in the *t*-test and the Chi-square test (*P* > 0.05). As shown in Table 1.

### 3.2. Comparison of Surgical Conditions

The length of hospital stay and VAS score in the treatment group were significantly lower than those in the control group, and the operation time and intraoperative bleeding were significantly higher than those in the control group, with statistically significant differences (*P* < 0.05). While the success rate of the one-sided operation was 86% higher in the treatment group than 84% higher in the comparison group, the statistical comparison was not statistically significant (*P* > 0.05)(Figure 1).

### 3.3. Comparison of Inflammatory Factor Levels

There was no statistically significant difference (*P* > 0.05) in the comparison of inflammatory responses between the two groups of children before surgery, while the comparison of CRP, IL-6, and calcitoninogen between the two groups of children after surgery was significantly different and lower in the comparison group than in the treatment group, and the statistical comparison was statistically significant (*P* < 0.05). (Figure 2).

### 3.4. Clinical Efficacy

The clinical efficacy of the two groups showed that the incidence of complications such as urinary fistula, urethral stricture, and urethral diverticulum, and urethral rupture in the treatment group was 16.00%, which was significantly higher than that in the control group (4.00%), and the difference was statistically significant (*P* < 0.05)(Figure 3).

## 4. Discussion

In recent years there has been a growing interest in the long-term outcome of hypospadias, with a particular focus on postoperative penile appearance, and staging has once again returned to the mainstream [8]. It is more widely recognised that passive use of an inadequate foreskin flap to complete a stage I hypospadias correction will increase the risk of complications and sacrifice penile appearance [9]. Therefore, a planned and proactive staging option is a reasonable decision, especially in the case of heavy hypospadias, where the choice may not be between staging and staging, but between active and passive staging [10]. If there is a planned choice of the staged surgery, the requirements of its first phase should not be limited to some specific corrective elements, but should be understood as creating good corrective conditions for the second phase of surgery [11]. In addition to completely correcting the hypospadias, the first stage of surgery allows for partial reconstruction of the urethra where appropriate, reducing the length of the urethra repaired during the second stage, and reducing the risk of each stage of the surgery [12]. Although conventional staged surgery can address the problem of insufficient flaps, the new urethra to be repaired at the second stage is longer and prone to postoperative urethral fistula or urethral stricture [13]. Early surgeons commonly used traditional staged surgery as follows: transection of the urethral plate in the first stage to completely correct the hypospadias, and repair and reconstruct the urethra in the second stage to reshape the appearance of the penis [14]. However, with the accumulation of surgical experience and progressive research into the treatment of hypospadias, the one-stage surgery for hypospadias began to take shape [15]. The concept and method of staged surgery for hypospadias is becoming accepted worldwide, and as specialisation in hypospadias continues to advance, the technique of staged surgery is becoming more sophisticated and is superior to staged surgery in terms of complications, number of operations, difficulty, and psychological impact on the child [16]. Staged surgery has become the treatment of choice for a few very heavy cases or in less technologically advanced areas, and the concept of staged urethral reconstruction is gradually being phased out of clinical practice [17]. Staged surgery means balancing the difficulty and risk of surgery in each stage in order to reduce the difficulty of the operation and the incidence of postoperative complications in each stage, so as to better achieve the orthodontic goals and obtain the most satisfactory penile appearance, based on the premise of achieving the goals of hypospadias treatment: near-normal appearance, straight penis, orthodontic opening, normal urinary flow, and urinary line, and low complication rate [18].

This study explored the Duckett procedure, which is a transfer of the tipped insular inner foreskin plate flap to the ventral side as a modification of the previous procedure, severing the urethral plate to completely straighten the penis. The inner foreskin plate is ideal for urethral repair and reconstruction. It has sufficient skin, easy access, high survival rate of the tipped flap, resistance to urinary irritation, abundant blood flow, and proximity to the urethral orifice, and the combination of multilayered tissue coverage and staggered sutures can effectively reduce the incidence of urethral fistula after hypospadias [19]. The results showed that the length of hospital stay and VAS score of children in the treatment group were significantly lower than those in the comparison group, while the operative time and intraoperative bleeding were higher in the treatment group than those in the comparison group, and the success rate of one operation was higher than that of the comparison group. The Duckett procedure takes full advantage of the physiological and anatomical features of the foreskin to make the penis look like a circumcision after surgery, and the Duckett procedure ensures that postoperative contracture of the duct is reduced and the success rate of the operation is improved [20]. The common complication of the Duckett procedure is urethral fistula, but the method of repair is relatively simple and has a high success rate [15]. The disadvantage of the procedure is that it is complex, requires a high level of surgical skill, and requires more experience to achieve a satisfactory outcome [21]. The differences in CRP, IL-6, and calcitoninogen between the two groups were statistically significant and lower in the comparison group than in the treatment group. CRP is an important indicator of inflammation and its synthesis rises rapidly as a response to inflammatory stimuli and is an early sensitivity to infection [22].

The Duckett procedure is a one-stage repair of hypospadias that allows complete straightening of the inferior penile curvature and easy access to the material [23]. However, if the indications for the staged Duckett surgery are not strictly understood, the success rate will be reduced and the incidence of postoperative complications will be increased. Only by strictly understanding the indications for the staged Duckett surgery and making a reasonable choice can clinicians improve the success rate and reduce complications [22]. The success rate of the staged Duckett surgery is higher than that of staged Duckett surgery, and the choice of the staged Duckett surgery is likely to improve the outcome of the procedure [24]. This is because the staged Duckett surgery is a better solution to the shortage of local repair material, shrinkage of the original urethral plate scar, and poor blood supply encountered during a one-stage Duckett repair [25]. It also reduces the risk of complications and achieves a better penile appearance, particularly in cases of severe hypospadias complicated by penile dysplasia [26]. The risk of postoperative complications is increased if the surgeon does not assess the local anatomy of the penis in a planned way before surgery and blindly chooses to perform a one-stage procedure [27]. Passive second-stage surgery, or even multiple surgeries, can result in residual penile hypospadias and local skin scar contracture, and this “passive” staging can lead to more difficult, longer, and more costly repairs, and can even leave a deformed penile appearance [28]. It has been suggested that second-stage surgery results in a more aesthetically pleasing penile appearance and no significant increase in complications compared to first-stage surgery [29]. This is also true of the domestic data, where the active and planned choice of the staged Duckett surgery has a lower incidence of major postoperative complications than the stage I Duckett surgery; therefore, we can assume that staged surgery for severe hypospadias and hypospadias that has undergone multiple surgeries has satisfactory clinical outcomes [30].

Urethral fistula is the most common complication of hypospadias surgery and is the main reference factor in evaluating the success or failure of the procedure. Poor blood supply to the formed urethral extraction, local tissue ischaemia, necrosis, and infection are the main causes of postoperative urethral fistula [31]. There are also cases where poor drainage of urine due to the urethral stricture increases the tension of the incision, causing it to split and form a urinary fistula [32]. We need to fully understand the characteristics of the vascular distribution of the foreskin; the vascular tip should be free and wide as possible, the anatomical level should be clear and distinct to avoid damaging its vascularity, and the rich blood supply can easily make the newly formed urethra heal and can enhance the resistance of the tissue to infection [33]. This can lead to poor healing of the incision after surgery, resulting in urethral fistula [34]. The development of postoperative urethral fistula complications, especially if multiple surgeries are performed due to complications, can have long-term physical and psychological effects on the patient [35]. Urethral stricture is also a common postoperative complication of hypospadias, usually occurring around 12 months after urethroplasty, and can occur in the early postoperative period [36]. The causes of urethral stricture are multiple and complex and are mainly related to postoperative infection, flap scar contracture, and a small flap design that does not match the size of the penis; therefore, the flap should not be designed to be too small during surgery, otherwise, combined with conditions such as flap contracture, the newly formed urethra will be narrow [37]. Although the results of this study showed no statistical difference in the incidence of urethral strictures between the two groups, urethral strictures are also a common complication of both procedures and can occur in all segments of the neourethra. Urethral strictures are more common at the anastomosis of the neourethra and the original urethra, where a beveled anastomosis is performed to reduce the occurrence of anastomotic strictures, but they are still difficult to avoid. In addition to the aforementioned factors, urethral strictures are also associated with damage to the urethral corpus cavernosum during the beveled anastomosis of the neourethra and the original urethra, which can lead to scarring of the anastomosis and result in anastomotic strictures [38].

The present study is novel but deficient in which the clinical efficacy of the Duckett procedure for hypospadias is significant, but the exact mechanism has not been studied in depth over time. The collection of cases from the same hospital was poorly representative and the exclusion and inclusion criteria were subjective, which may have led to biased results.

In conclusion, the staged Duckett procedure is clinically more effective than the one-stage Duckett procedure, with a higher success rate and lower complication rate. It is able to break down a complex procedure into two relatively simple operations, the technical requirements and risk of failure of the first-stage procedure are greatly reduced, and it is significantly more effective in reducing the patient's major postoperative urethral fistula, urethral stricture, urethral disintegration, and penile recurvature. The first stage of the procedure has a much lower technical requirement and risk of failure. It is worthwhile to promote the use of this procedure in clinical practice as it has a more aesthetic penile shape and functional results.

## Figures and Tables

**Figure 1:** Surgical situations of the children in the two groups (hospital stay, operative time, vascular score, and intraoperative bleeding) were expressed as mean ± standard deviation (*X* ± *S*) and calculated by the *t*-test. The success rate of one operation was expressed as an integer using the chi-square test for the count data. The results showed that the length of stay and VAS score of the children in the treatment group were significantly lower than those in the comparison group, while the operation time and intraoperative bleeding were higher than those in the comparison group, and the statistical comparison was statistically significant (*P* < 0.05). While the success rate of the primary surgery was 86% higher in the treatment group than 84% higher in the comparison group, the statistical comparison was not statistically significant (*P* > 0.05).

**Figure 2:** Comparison of inflammatory responses between the two groups (CRP, IL-6, and procalcitonin and other indicators were expressed as mean ± standard deviation (*X* ± *S*) using *t*-test, and the success rate of one operation was expressed as an integer using chi-square test The results showed that there were significant differences in CRP (a) IL-6 (b), and procalcitonin (c) between the two groups after surgery, and the comparison group was lower than the treatment group, The comparison is statistically significant (*P* < 0.05)).

**Figure 3:** Comparison of complications between the two groups of children (the enumeration data of the clinical efficacy of the two groups of children were analyzed and expressed as integers. The incidence of complications such as urethral fistula, urethral stricture, urethral diverticulum, and urethral rupture was significantly higher than that of the control group (4.00%, 16.00%), and the difference was statistically significant (*P* < 0.05)).

**Table 1:** Comparison of general information between the two groups (*n*, $\bar{x}\pm s$).

Groups	Average age (years)	Body mass index (kg/m^2^)	Width of the urethral plate (cm)	Degree of penile curvature		
				Coronal sulcus	Penile corporis	Penile scrotum
Comparison group	6.78 ± 1.32	23.78 ± 3.32	0.34 ± 0.05	14	25	11
Treatment group	6.62 ± 1.66	23.62 ± 3.66	0.31 ± 0.04	13	27	10
*χ* ^2^/*t*	0.533	0.229	0.113	0.051	0.160	0.060
*P*	0.595	0.819	0.992	0.822	0.689	0.806

## Data Availability

The datasets used and analyzed during the current study are available from the corresponding author upon reasonable request.
